The article "Application of Dynamic Process Neural Network Model Identification in Ethnic Dance Online Teaching System" was published in 2022. Journal: Comput Intell Neurosci.

# Application of Dynamic Process Neural Network Model Identification in Ethnic Dance Online Teaching System

**DOI:** 10.1155/2022/2825530

**Published:** 2022-07-13

**Authors:** Jun Hu, Tianshi Hou

**Affiliations:** Hebei Normal University Huihua College, Shijiazhuang, Hebei 050091, China

## Abstract

With the development of the times, education presents a new trend, but the teaching characteristics of dance classroom teaching cannot adapt to the current development trend. In this article, the author analyzes modern information technology, hoping to realize the teaching of folk dance on the Internet and provide a new model of online distance teaching for folk dance teaching. The author analyzes the current teaching problems in colleges and universities, and proposes to change the existing teaching situation based on dynamic process neural network model identification and artificial intelligence, and instead use online remote network ethnic dance teaching. Online distance education can enable flexible teaching of folk-dance courses, deeply dig into the theoretical basis of distance teaching, and use online distance network teaching to make teaching time more flexible, not only providing new teaching methods but also introducing new teaching concepts. Based on the traditional neural network model identification, a dynamic process neural network model identification is developed. This model is no longer subject to the input limitation of the traditional neural network model, the processing time is relaxed, and the advantages are more obvious. In this research, the author introduces dynamic process neural network model identification in time series data mining, and makes full use of artificial intelligence to deeply analyze the classification and prediction problems in the context of time series.

## 1. Introduction

Different from other traditional courses, dance is a comprehensive course, artistic, so it is different from other courses in teaching mode [1]. In the process of dance teaching, teachers often need to explain the theoretical content verbally. Teachers should personally demonstrate some difficult content, give students correct examples, and combine theory with teaching [2]. Under the guiding ideology of system science, teachers must make reasonable arrangements for the entire teaching process, carefully analyze the content of the professor, and fully understand the mastery and physical conditions of each student [3]. In the teaching process, the teacher should actively solve the problems raised by the students, arrange the teaching content according to the teaching materials, and all teaching activities should be carried out around the teaching materials. To attract students' interest, teachers should carefully design courses during the teaching process, set up suspense for certain issues, enable students to actively explore based on curiosity, and allow students to participate more actively in learning, which will help promote teaching Integration [4]. In the process of social development, the role of artificial intelligence has become more and more prominent. Artificial intelligence has been applied to various fields, and while exerting advantages in various fields, there are also certain problems [5]. Nowadays, artificial intelligence has been applied in the field of education, and robots have also appeared in the field of dance teaching [6]. In this article, we deeply analyzed the artificial intelligence teaching technology and studied the characteristics of the dance discipline and the characteristics of this profession. In this article, we use the literature review method to analyze the role of artificial intelligence in the process of dance teaching, analyze the advantages and disadvantages of artificial intelligence, and hope that it can provide reference suggestions for the development of artificial intelligence in the field of dance teaching.

The article "Application of Dynamic Process Neural Network Model Identification in Ethnic Dance Online Teaching System" was published in 2022. Journal: Comput Intell Neurosci.

## 2. Related Work

Some research studies the basic ideas of college dance teaching mode, analyzes the actual situation of college teaching, and judges the requirements of colleges on the dance teaching system [7]. Follow the software engineering design ideas and advanced development concepts to develop the system and set up reasonable functional sections. The literature establishes a complete remote online system development template through programming language [8]. Some research studied the framework structure of the online dance teaching system based on the application of software engineering ideas and database technology, analyzed the function of each module in the system according to the requirements, designed the application interface of the system, and determined which should be used Data transmission algorithm [9]. Some research tests each module of the online dance teaching system that has been designed, and the test angles include memory occupancy rate, temperature, and CPU occupancy rate, and then analyzes whether the functions of the remote online dance teaching system can meet the user's needs demand [10]. Some research analyzes the teaching system in the research, uses modern programming methods and database technology, analyzes the current shortcomings in teaching in colleges and universities, and analyzes the advantages of online remote dance teaching [11]. Using online remote dance teaching can make teaching More flexible. Nowadays, there are serious problems in dance teaching. To solve this problem, a remote online dance teaching system was designed. In this system, teachers and students can interact [12]. The emergence of this system provides a new teaching model for dance teaching and enriches teaching methods. Some research uses a lot of video data in the process of dance teaching [13]. To solve the problem of data presentation, in this article, the author uses signal encoding and decoding algorithms to process the data and completes the video by encoding and decoding. During the use of the remote online dance teaching platform, teachers need to upload various video materials, and students should download video materials according to their own needs. In the process of uploading and downloading, the system must judge the legality of the video, and analyze whether the video meets the scope of the dance teaching video according to the content of the video [14]. In this article, we use dynamic process neural network model identification and artificial intelligence technology to enrich the learning methods of the nation [15].

The article "Application of Dynamic Process Neural Network Model Identification in Ethnic Dance Online Teaching System" was published in 2022. Journal: Comput Intell Neurosci.

## 3. Dynamic Process Neural Network Model Identification Model Identification

### 3.1. Dynamic Process Neural Network Model Identification Model

The structure of the process neuron is composed of three parts: aggregation, weighting, and excitation operation. The difference between it and the traditional neuron is that the input, output, and corresponding weight of the process neuron are all time-varying, and its aggregation operation includes both the multi-input aggregation of the space and the cumulative aggregation of the time process. The structure diagram of a single process neuron is shown in Figure 1. Figure 1 includes linear functions, Sigmoid functions, Gauss-type functions, etc.

Process neural network model identification is a network type, and its composition follows a certain topological structure.  Figure 2 is a topological structure identified by a process neural network model. The output value of this structure is a constant.

Process neural network identification is a feedforward process neural network model. Both the output value and the input value are time-varying functions. In the network, the input and output relationship between each layer is as follows:

System input:

(1) $$\begin{array}{c} X\left(t\right)=\left(x_{1}\left(t\right),x_{2}\left(t\right),\ldots ,x_{n}\left(t\right)\right). \end{array}$$

The first hidden layer output:

(2) $$\begin{array}{c} y_{j}^{\left(2\right)}=f_{1}\left(\sum_{i=1}^{n}\int_{0}^{T}w_{ij}\left(t\right)x_{i}\left(t\right)\text{d}t-\theta_{j}^{\left(1\right)}\right),\;j=1,\Lambda ,m. \end{array}$$

The second hidden layer output:

(3) $$\begin{array}{c} y_{l}^{\left(2\right)}=f_{2}\left(\sum_{j=1}^{m}v_{jl}y_{j}^{\left(1\right)}-\theta_{l}^{\left(1\right)}\right),\;j=1,\Lambda ,m\;l=1,\Lambda ,L. \end{array}$$

The output layer looks like this:

(4) $$\begin{array}{c} y=\sum_{l=1}^{L}y_{l}^{\left(2\right)}\mu_{l},\;l=1,\Lambda ,L. \end{array}$$

After bringing into the model, the input and output relationship between the layers of the network is:

System input:

(5) $$\begin{array}{c} X\left(t\right)=\left(x_{1}\left(t\right),x_{2}\left(t\right),\ldots ,x_{n}\left(t\right)\right). \end{array}$$

The first hidden layer output:

(6) $$\begin{array}{c} y_{j}^{\left(1\right)}=f_{1}\left(\sum_{i=1}^{n}\int_{0}^{T}w_{ij}\left(t\right)x_{i}\left(t\right)\text{d}t-\theta_{j}^{\left(1\right)}\right),\;j=1,\Lambda ,m. \end{array}$$

The second hidden layer output:

(7) $$\begin{array}{c} y_{l}^{\left(2\right)}=f_{2}\left(\sum_{j=1}^{m}v_{jl}y_{j}^{\left(1\right)}-\theta_{l}^{\left(1\right)}\right),\;j=1,\Lambda ,m\;l=1,\Lambda ,L. \end{array}$$

To meet the requirements of the expansion coefficient range of the output function orthogonal basis, the output layer is as follows:

(8) $$\begin{array}{c} y=\sum_{l=1}^{L}y_{l}^{\left(2\right)}\mu_{l},\;l=1,\Lambda ,L. \end{array}$$

When processing information, it must be done in order. The output of the first-level nodes will not affect the output of the upper-level nodes, and there is no feedback between different levels. The feedback process neural network model identification model contains a total of 3 layers. In the input layer, the time-varying process signal of the system can be input, the output signal of a neuron can be output, and the output result can be fed back to the input layer. The spatiotemporal aggregation operation of the hidden input signal is completed in the output layer. Since the network weight function is arbitrary, the orthogonal basis function should be selected in the input space, which is a problem of training the coefficients of the weight function.

The article "Application of Dynamic Process Neural Network Model Identification in Ethnic Dance Online Teaching System" was published in 2022. Journal: Comput Intell Neurosci.

In the input layer of the network, the time-varying process input of the network depends on nodes to complete, and the information output by the contacts must be fed back to the system. In the process of neuron, the number of nodes in the hidden layer is different from that of the input layer. The output of information, feedback to the input layer, and spatial aggregation operations can all be done through nodes. The spatiotemporal aggregation operation of the output signal can be completed by the process neuron in the input layer.

The output of the hidden layer of the process neuron is given by:

(9) $$\begin{array}{c} u_{j}\left(t\right)=f\left(\sum_{i=1}^{n}\left(w_{ij}\left(t\right)\left(x_{i}\left(t\right)+\sum_{j=1}^{m}w_{ij}\left(t\right)u_{j}\left(t-\tau \right)\right)\right)\right). \end{array}$$

The corresponding output of the neural network model identification in the feedback process is given by:

(10) $$\begin{array}{c} y=g\left(\int_{0}^{T}\left(\sum_{j=1}^{m}v_{j}\left(t\right)u_{j}\left(t\right)\right)\text{d}t-\theta \right). \end{array}$$

The calculation process of process neural network model identification is different from the calculation of traditional network neural model identification. There will be many basis functions in the function space. In the calculation process of process neural network model identification, to avoid repeated calculations, When choosing an orthogonal basis function, the conditions that the function should satisfy are as follows:

(11) $$\begin{array}{c} \int_{a}^{b}f\left(x\right)g\left(x\right)\text{d}x=0. \end{array}$$

According to the needs of users, orthogonality should be transformed into weighted orthogonality:

(12) $$\begin{array}{c} \int_{a}^{b}h\left(x\right)f\left(x\right)g\left(x\right)dx=0. \end{array}$$

Under normal circumstances, the orthogonal basis functions that people use are as follows:

(1) Triangular basis function
(2) The most commonly used in the orthogonal function system is the trigonometric function system:
  (13) $$\begin{array}{c} \left\{\frac{1}{\sqrt{2\pi }},\frac{1}{\sqrt{\pi }}\cos\;x,\frac{1}{\sqrt{\pi }}\sin\;x,\frac{1}{\sqrt{\pi }}\cos\;2\;x,\frac{1}{\sqrt{\pi }}\sin\;2\;x,\ldots ,\frac{1}{\sqrt{\pi }}\cos\;nx,\frac{1}{\sqrt{\pi }}\sin\;nx,\ldots \right\}. \end{array}$$
(3) Orthogonal polynomial

In addition to polynomial functions:

(14) $$\begin{array}{c} \text{0}<\int_{a}^{b}h\left(x\right)\text{d}x<+\infty . \end{array}$$

If the interval is infinite, the following formula must converge:

(15) $$\begin{array}{c} h_{n}=\int_{a}^{b}x^{n}h\left(x\right)\text{d}x,\;\left(n=0,1,2,\ldots \right). \end{array}$$

The following conditions need to be met:

(16) $$\begin{array}{c} \int_{a}^{b}h\left(x\right)P_{m}\left(x\right)P_{n}\left(x\right)\text{d}x=0,\;\left(m\neq n\right). \end{array}$$

Recorded as:

(17) $$\begin{array}{c} \left\|P_{n}\right\|=\sqrt{\int_{a}^{b}h\left(x\right)P_{n}^{2}\left(x\right)\text{d}x}. \end{array}$$

For example, each formula must meet the following conditions:

(18) $$\begin{array}{c} \left\|P_{n}\right\|=1. \end{array}$$

Appropriate orthogonal basis functions are introduced in the process neural network model identification, and this function is usually standard. Expand the orthogonal function, and the equation obtained is the input function. In addition, the expansion of the same orthogonal basis function can be used as the weight function of the time-varying process neuron hidden layer. After considering the orthogonality of basis functions, process neural network model identification, the complexity of construction operation is greatly reduced, and the amount of calculation required is also greatly reduced. Practice shows that using this method can make the network more stable and improve the convergence rate of the network. Under this premise, the feedback process, the learning process of the neural network and the training process of the traditional feedforward neural network model identification are all equally complex.

The article "Application of Dynamic Process Neural Network Model Identification in Ethnic Dance Online Teaching System" was published in 2022. Journal: Comput Intell Neurosci.

### 3.2. Self-Organizing Process Neural Network Model Identification

In the process of process neural network model identification and calculation, it is necessary to introduce standard orthogonal basis functions. When inputting the function, expand the orthogonal basis function. To make it easier for the process neural network model to identify space-time operations, the author uses the orthogonality of the product function. Through experiments, we know that using this method can greatly improve stability. In the learning process of neural networks, both the process neural network model and the feedforward neural network model require equally complex calculations.

The self-organizing process neural network model identification is used to solve the pattern classification problem related to the time process. To allow the unmarked sample information to be reasonably used, the author proposes a dynamic sample semi-supervised learning algorithm, which is developed based on the self-organizing process neural network model identification. In the self-organizing process of neural network model identification, there are only two hierarchical structures: one is the input layer, and the other is the competition layer.  Figure 3 shows the self-organizing process neural network model to identify the topological structure:

To minimize the amount of calculation, in this article, the orthogonal basis expansion method is used in the overall calculation of the network. In the transportation process, the first standard orthogonal basis function is introduced. According to the nature of the orthogonal basis function, the operation is transformed into a time-invariant problem.

Competitive learning algorithm,

**Definition 1 as:.**

(19) $$\begin{array}{c} \langle X\left(t\right),Y\left(t\right)\rangle ={\int_{0}^{T}X\left(t\right)\left(Y\left(t\right)\right)}^{T}\text{d}t. \end{array}$$

**Definition 2 .**

(20) $$\begin{array}{c} \left\|X\left(t\right)\right\|={\left(\langle X\left(t\right),Y\left(t\right)\rangle \right)}^{\left(1/2\right)}\\ ={\left({\int_{0}^{T}X\left(t\right)\left(Y\left(t\right)\right)}^{T}\text{d}t\right)}^{\left(1/2\right)}. \end{array}$$

**Definition 3 .**

(21) $$\begin{array}{c} r=\frac{\langle X\left(t\right),Y\left(t\right)\rangle }{\left\|X\left(t\right)\right\|\cdot \left\|Y\left(t\right)\right\|}. \end{array}$$

Based on mathematical analysis theory

(22) $$\begin{array}{c} x_{i}\left(t\right)=\sum_{l=1}^{L}a_{il}b_{l}\left(t\right),\;i=1,2\Lambda ,n,\\ w_{ii}\left(t\right)==\sum_{l=1}^{L}w_{il}^{\left(1\right)}b_{l}\left(t\right),\;i=1,2\Lambda ,n;\;j=1,2\Lambda ,m. \end{array}$$

Therefore, it has the following properties:

(23) $$\begin{array}{c} \int_{0}^{T}b_{l}\left(t\right)b_{s}\left(t\right)\text{d}t=\left\{\begin{array}{c} 0,\;l\neq s,\\ 1,\;l=s. \end{array}\right) \end{array}$$

The neuron that wins the competition is the node with the largest similarity coefficient, as shown below:

(24) $$\begin{array}{c} r_{j}{*}^{k}=\underset{j\in \left\{1,2,\Lambda ,m\right\}}{\max}\left\{r_{j}^{k}\right\}. \end{array}$$

Dynamic process analysis is a perfect combination of functional analysis, Fourier analysis, harmonic analysis and numerical analysis. Process dynamic analysis is a branch of mathematics with strong applications. It can be used in many fields, such as signal processing, voice recognition, diagnosis of fault analysis, stock market conditions, and image processing. Using process dynamic analysis, you can have a more detailed understanding of the analyzed content. For the low-frequency part of some signals, dynamic process analysis can be used to make the time resolution lower without reducing the frequency resolution. In this article, we are forced to use dynamic process technology to decompose and reconstruct discrete dynamic processes. The author combines the characteristics of time series data processing to analyze the decomposition and reconstruction of discrete dynamic processes.

The article "Application of Dynamic Process Neural Network Model Identification in Ethnic Dance Online Teaching System" was published in 2022. Journal: Comput Intell Neurosci.

### 3.3. Experimental Results and Analysis

To analyze whether the above method is effective, cluster analysis is performed using the initial value of the randomly given weight function. The final comparison result is shown in Table 1:

According to the above experiment, using the same training sample and experimental sample, the method used in this article and the method proposed in the literature are tested and the results are compared. The final result comparison is as follows:

According to the data in Table 1 and 2, the method proposed in this article is compared with the method in the literature. Through the experimental results, it can be found that the method used in this article is far more accurate than the method proposed in the literature and has lower accuracy. The number of runs requires less running time. For the algorithm of this article, the author analyzes the algorithm from two aspects: the quality of clustering and the speed of clustering. Through analysis and other quality, we can judge the accuracy of clustering of the algorithm used in this article. Through a large number of experiments, it can be known that the accuracy of clustering of the algorithm used in this article is still high under different sample sizes. In the case of different sample sizes, use the algorithm provided in this article and the algorithm in the literature to cluster the numbers, and the final result is shown in the above formula. When the number of samples increases, the amount of time required for each algorithm will increase accordingly. If the clustering is based on a certain number of samples, the algorithm provided in this article will take less time than the algorithm in the literature. This is because the initialization method and weighted Euclidean distance formula are used in this article to improve the convergence speed of the network, greatly reduce the running time, and have better performance. Clustering accuracy as shown in Table 3.

To make the online dance teaching system better meet the needs of users, it is necessary to confirm the users of the system, such as students, teachers, administrators, etc. Different users have different expectations of the system, and the permissions they have after logging into the system are different. For example, the administrator in the system should assume the responsibility of managing data, such as the data uploaded by the teacher, the account that the teacher logs in, the account that the student logs in, and so on. Teachers can upload materials and issue homework in the system, while students can log in to the system, download the materials uploaded by the teacher, and complete the homework assigned by the teacher. In the system test stage, if any teacher or student thinks that the functions in the system are not perfect, they can apply to the Academic Affairs Office. After review by specialized personnel, if the application is determined to be reasonable, they can open this function. Conducive to the system to better serve students and teachers and meet the needs of teaching. Normally, the remote online dance teaching system must be composed of three users: teacher, administrator, and student. Therefore, in this article, the author analyzes the functions of these three and the requirements for system functions.

## 4. Design of an Online Teaching System for Ethnic Dance Based on Artificial Intelligence

### 4.1. Video Teaching Subsystem

In online dance distance teaching, the teacher is the most important role and a full participant. Teachers should log in to the system to explain and demonstrate dance movements, arrange students' learning tasks, guide students' movements, answer any questions that students have during training, and upload some important video materials to assist students in learning. According to the teaching process, the teacher needs to upload the teaching courseware, as well as the required teaching video pictures and other materials, the teacher must reasonably configure the teaching materials, use a reasonable teaching method, and supervise the students to learn. In the remote teaching system, teachers must upload courseware in time, upload teaching resources in time, assign homework in time, and regularly interact with students to answer student questions and so on.

The article "Application of Dynamic Process Neural Network Model Identification in Ethnic Dance Online Teaching System" was published in 2022. Journal: Comput Intell Neurosci.

#### 4.1.1. Teacher

In the online dance distance teaching, the teacher is the most important role and a full participant. Teachers should log in to the system to explain and demonstrate dance movements, arrange students' learning tasks, guide students' movements, answer any questions that students have during training, and upload some important video materials to assist students in learning. According to the teaching process, the teacher needs to upload the teaching courseware, as well as the required teaching video pictures and other materials. The teacher must reasonably configure the teaching materials, use reasonable teaching methods, and supervise the students' learning. In the remote teaching system, teachers must upload courseware in time, upload teaching resources in time, assign homework in time, and regularly interact with students to answer student questions and so on.

#### 4.1.2. Students

Online dance distance teaching system, but the ultimate goal is to provide services for students. Whether the system has met the needs of students for learning dance courses can be understood through students' evaluation and description of the system. Students log in to the online dance distance teaching system and ask questions through the communication platform. To solve the problem, download the uploaded materials in time and complete the homework assigned by the teacher. Students should log in to the remote education system in time to complete course testing and teaching quality evaluation.

#### 4.1.3. Administrator

Administrators play an important role in the online distance dance teaching system. When the system is running normally, the administrator must maintain and manage the system. When there is a problem in the system, the administrator must solve the problem in time. The administrator should adjust the system in response to the feedback from teachers and students on the website on time. When more and more people use the system, more and more opinions are put forward for the system, which is conducive to improving the system and perfecting the functions of the system, and it is also conducive to the learning and use of students. In the remote teaching system, the administrator must save the information of teachers and students, build a communication forum, and update it in time. The upload and download status of teachers and students must be managed by the course selection and lesson plan. It is necessary to record the running status of the system and students' course grades. Through the analysis of system users, we can understand the needs of each system user, and then set the functions of the system. The functions of each module in the online dance teaching system are shown in Figure 4:

The article "Application of Dynamic Process Neural Network Model Identification in Ethnic Dance Online Teaching System" was published in 2022. Journal: Comput Intell Neurosci.

### 4.2. Teacher-Student Interaction Subsystem

In the online dance system, teachers and students have different permissions and can perform different functions. Teachers mainly upload courseware and materials while students mainly download materials and complete homework. The specific functions are shown in Figure 5. Through positive incentives, administrators can have a positive influence on teachers and class leaders, and teachers and class leaders can further influence students. Such influence is called positive influence. Teachers or class leaders influence administrators, and teachers and class leaders will be influenced by students. This kind of influence is called “negative feedback.” “Negative feedback” will also have a certain impact on the development of work, which is conducive to gaining experience from teachers and students and improving work. Students will grade the courses of each semester and will also evaluate the content taught by the teacher, which will play a supervising role for the teacher. Through one semester of study, teachers and students can also evaluate the system, which is helpful for the administrator to modify and manage the website. Some students reported in the system that only videos are allowed to be downloaded, not pictures. Some students want to download a certain action picture, which cannot be achieved, so they hope that the system can add this function, and the addition of the function requires the administrator's background operation. For teachers, if the speed of uploading the video is too slow, you can upload the action image first, and then upload the entire video to the system. Users of each system can improve the system through feedback to meet their own needs. In this way, whether it is teaching work or system management, it will play a certain incentive role. With the continuous improvement of the system, it will help promote the popularization of distance education and teaching. The relationship between teachers, class leaders, students, and administrators is shown in Figure 5.

The article "Application of Dynamic Process Neural Network Model Identification in Ethnic Dance Online Teaching System" was published in 2022. Journal: Comput Intell Neurosci.

Table 4 shows the process of how to upload video materials, pictures, files, and courseware on the teacher side.

Table 5 shows the process of teachers assigning homework.

### 4.3. System Modeling Design

The use of video compression algorithms does not pay attention to how the bytes are sealed by the media on the platform but only cares about how to convert the video into a byte data stream. If you analyze the method in the traditional sense: this compression method is a destructive data compression method. When compressing video, all compressed images will cause quality damage. Based on the IPEG video compression algorithm, a new compression algorithm is formed. The compression form of this algorithm is lossless, but it is not widely used. The data after the image and video compression format can be integrated into other file formats.

The most common way to store pictures on the World Wide Web and transfer pictures is the JPEG video compression algorithm. This algorithm does not rely on drawing marks and text icon graphics at all. Because the use of this compression method is not the best for these image compression formats and can hardly get satisfactory results, we think this method is not suitable for storing some color images or color videos.

There are a variety of MPEG video compression algorithms, including MPEG1, MPEG2, MPEG4, MPEG7, and MPEG21. The first four letters of these compression algorithms are the same, that is, the numbers that follow are different. A group that has developed MPEG video compression algorithms, specializing in image and video compression methods. MPEG will cause certain damage to the compressed content when compressing various video formats. The main working principle is as follows: through the sampling amplifier, the optical signal is formed into a video signal. In this case, the video signal is regarded as an image, and the image is divided into various parts. Each part is a specific area. In the region, the content on the image is transformed and encoded, and then the entire image is encoded, so that the compression process is completed.

## 5. Conclusion

With the advancement of technology, digitalization has become a trend of the times. Computers and digital media are used in our study, work, and entertainment life. The pace of information digitization is getting faster and faster, and almost every industry has been affected by digitization. Dance education is a highly artistic education. When digitalization is integrated into the dance education process, the laws of dance art should be studied. When applying digitization to subjects with artistic flavor, it is necessary to understand the common ground of information between technology and art and develop and research the digitization of dance teaching on this basis. In every professional field, the system must be scientifically researched. In this paper, the dynamic process, neural network model recognition, and artificial intelligence methods are analyzed to study the problems existing in online dance education. It is necessary to discuss in depth the dynamic process of neural network model recognition and artificial intelligence to make it better applied to dance education. The problems existing in the online dance teaching system must be solved in time, and the technical staff must develop the system reasonably and expand related work, rationally allocate resources, and integrate projects.

The article "Application of Dynamic Process Neural Network Model Identification in Ethnic Dance Online Teaching System" was published in 2022. Journal: Comput Intell Neurosci.

## Figures and Tables

**Figure 1:** Process neuron.

**Figure 2:** A forward process neural network model to identify topological structure.

**Figure 3:** Self-organizing process neural network model to identify topological structure.

**Figure 4:** Functions of each sub-module in the online dance teaching system.

**Figure 5:** Distribution diagram of the relationship among teachers administrators, monitors and students.

**Table 1:** Comparison of the results of different initial values.

Initialization method	Correct rate (%)	Number of runs	Running time (s)
Method of this article	93.33	5	25
Randomly given method	83.33	12	49

**Table 2:** Comparison of results of different clustering methods.

Clustering method	Correct rate (%)	Number of runs	Running time (s)
Method of this article	93.33	5	25
Comparison method	80.00	63	132

**Table 3:** Clustering accuracy.

Clustering	True clustering	The algorithm in this paper	Accuracy (%)
C1	16	13	81.25
C2	16	14	87.5
C3	16	16	100
C4	16	16	100
C5	16	16	100
C6	16	16	100

**Table 4:** Management instructional video program execution process description.

Teacher assigns coursework	
Staff composition	Teacher, online distance dance teaching system.

Demand	The teacher enters the system after entering the user name and password to complete the upload of videos, data, homework, and courseware.

Operation process	1. The teacher enters the account and password to enter the system.
	2. Follow the prompts and system guide to enter the courseware management and upload interface.
	3. The teacher uploads the courseware, pictures, videos and other materials used in class to the system in advance, waiting for the administrator to review.
	4. Post the courseware according to the prompts and wait for review.
	5. Manage and maintain the system in accordance with system requirements.

Actual process	Teachers can view all the courseware that has been uploaded successfully or pending review, and summarize and classify the materials that have been successfully uploaded.

The article "Application of Dynamic Process Neural Network Model Identification in Ethnic Dance Online Teaching System" was published in 2022. Journal: Comput Intell Neurosci.

**Table 5:** Description of the execution process of the teacher's course assignment program.

Teacher assigns coursework	
Participant	Online teaching system for teachers, students, and distance dance courses.

Demand	The teacher logs in to the system through the user name and password and uploads materials through the prompts and function modules on the system page.

Operation process	1. The teacher enters the password and account to log in to the system.
	2. Follow the system prompts to enter the job layout interface.
	3. The teacher can put the prearranged exercises into the current homework list interface.
	4. Assign homework according to the course progress and open the download permission.

Actual process	Integrate and classify all kinds of jobs, view all jobs in the list.

## Data Availability

The data used to support the ﬁndings of this study are available from the corresponding author upon request.
